This article has been retracted.

# Longitude Variation of the microRNA-497/FGF-23 Axis during Treatment and Its Linkage with Neoadjuvant/Adjuvant Trastuzumab-Induced Cardiotoxicity in HER2-Positive Breast Cancer Patients

**DOI:** 10.3389/fsurg.2022.862617

**Published:** 2022-05-11

**Authors:** Hui Liu, Xiaoyan Hu, Lingyun Wang, Tao Du, Jing Feng, Ming Li, Lei Liu, Xiaofang Liu

**Affiliations:** Hematology and Oncology Department, The First People’s Hospital of Guiyang, Guiyang, China

**Keywords:** microRNA-497, fibroblast growth factor 23, neoadjuvant/adjuvant, trastuzumab induced cardiotoxicity, HER2-positive breast cancer

## Abstract

**Purpose:**

MicroRNA-497 (miR-497) is previously reported to target fibroblast growth factor 23 (FGF-23) and regulates cardiac injury, while their value in predicting drug-induced cardiotoxicity is not reported. Thus, the current study aimed to investigate the correlation of miR-497/FGF-23 with neoadjuvant/adjuvant trastuzumab-induced cardiotoxicity in human epidermal growth factor receptor 2 (HER2)-positive breast cancer patients.

**Methods:**

A total of 97 HER2-positive surgical breast cancer patients who received neoadjuvant/adjuvant trastuzumab contained regimens were enrolled; then, their peripheral blood mononuclear cells (PBMC) and serum were collected at baseline, after neoadjuvant treatment, at 3 months (M3), 6 months (M6), 9 months (M9), and 12 months (M12) after surgery. The PBMC was used for miR-497 measurements, and the serum was used for FGF-23 measurements. The cardiotoxicity events and incidence were recorded.

**Results:**

A total of 24 (24.7%) patients occurred cardiotoxicity during the treatment period. MiR-497 decreased from baseline (median: 0.955) to M12 after surgery (median: 0.602) (*p *< 0.001), while FGF-23 increased from baseline (median: 0.390 ng/mL) to M12 after surgery (median: 0.566 ng/mL) (*p *< 0.001); besides, the miR-497/FGF-23 axis greatly reduced from baseline (median: 2.545) to M12 after surgery (median: 1.222) (*p *< 0.001). At most time points, miR-497 was negatively related to FGF-23 (all *p *< 0.05). Notably, the miR-497/FGF-23 axis at all time points (including baseline, postneoadjuvant treatment, M3, M6, M9, and M12) was related to a lower risk of cardiotoxicity (all *p *< 0.05). Furthermore, the miR-497/FGF-23 axis was also positively correlated with the left ventricular ejection fraction (LVEF) at all time points (all *p *< 0.01).

**Conclusion:**

The MiR-497/FGF-23 axis serves as a potential indicator predicting trastuzumab-induced cardiotoxicity in HER2-positive breast cancer patients.

## Introduction

Breast cancer, as the most frequent malignancy diagnosed in females, takes up approximately 30% of the newly diagnosed malignancies annually among females, which also has been considered as the second most common cause of deaths from cancer among women globally (1–3). From the recent reports, approximately 18%–20% of breast cancer patients present with human epidermal growth factor receptor 2 (HER2) overexpression, and these patients are featured by rapid tumor progression, short remission period of chemotherapy, higher rate of recurrence, and poor disease-free survival and overall survival (4, 5). Hence, targeted therapy for HER2 has been a hotspot for breast cancer in recent years. Trastuzumab, a recombinant form of DNA humanized IgG monoclonal antibody, can selectively bind with P185 glycoprotein regulated by the HER2 gene on the cell surface, thereby blocking the downstream oncogenic signal pathways of tumor cells, inhibiting tumor cell proliferation and neovascularization (6, 7). However, trastuzumab has been reported to be associated with a high risk of cardiotoxicity, leading to cardiac dysfunctions such as heart failure in breast cancer patients (8, 9). Hence, a better understanding of the molecular mechanisms involving trastuzumab-induced cardiotoxicity will contribute to providing useful prognostic biomarker and therapeutic target for breast cancer therapy.

MicroRNA 497 (miR-497) plays a critical role in many human biological and pathological processes such as growth, metastasis, and angiogenesis (10–12). Previous data report that miR-497 may serve as a potential tumor suppresser in breast cancer through multiple mechanisms (including inducing apoptosis via targeting Bcl-w (10), interacting with miR-195 to inhibit cell proliferation and invasion (11), and suppressing cell growth via targeting SMAD7 (12)). Fibroblast growth factor 23 (FGF-23), a phosphaturic hormone involved in maintaining phosphate homeostasis, may also participate in tumorigenesis and tumor progression in breast cancer (13, 14). More importantly, both miR-497 and FGF-23 have been reported to regulate cardiosphere-derived cell (CDC) differentiation, mediate myocardial ischemia-reperfusion (I/R) injury, or affect myocardial hypertrophy in various cardiovascular diseases (15–17). Clinically, the miR-497/FGF-23 axis has been illustrated to predict attenuated major adverse cardiac and cerebral event (MACCE) risk in end-stage renal disease (ESRD) patients who underwent continuous ambulatory peritoneal dialysis (CAPD) (18). Based on the above mentions, we hypothesized that the miR-497/FGF-23 axis also affected cardiotoxicity in breast cancer patients, particular in HER2-positive breast cancer patients treated with neoadjuvant/adjuvant trastuzumab-involved regimens. However, the relevant information was still unclear. Hence, this study aimed to explore the correlation of the miR-497/FGF-23 axis with neoadjuvant/adjuvant trastuzumab-induced cardiotoxicity in HER2-positive breast cancer patients.

## Methods

### Subjects

Between January 2017 and May 2019, 97 HER2-positive breast cancer patients were consecutively recruited for this study. The main inclusion criteria were (1) pathologically confirmed breast cancer; (2) scheduled for receiving trastuzumab-contained regimens as neoadjuvant and adjuvant treatment; (3) female and age above 18 years; (3) Eastern Cooperative Oncology Group (ECOG) performance status (PS) of 0–1; (4) left ventricular ejection fraction (LVEF) ≥ 55% measured by echocardiography within 4 weeks before enrollment; (5) HER2 positive determined by immunohistochemistry (IHC) and further confirmed by fluorescence in situ hybridization (FISH); (6) no evidence of metastasis (M0); and (7) normal bone marrow, hepatic and renal function. The main exclusion criteria were (1) contraindications to drugs used in this study; (2) other malignancy within the last 5 years; (3) history of heart disease or insufficient cardiac function; (4) any concurrent disease that could affect compliance with the study protocol such as active infection, uncontrolled disease, organ allografts, and so on; (5) pregnant, lactating females, or women of childbearing potential without a negative pregnancy test; and (6) chronic daily treatment with aspirin and aspirin analogs or clopidogrel. Written informed consents were provided by all breast cancer patients. This study was approved by the Institutional Research Ethics Committee.

### Date Collection

Baseline characteristics of HER2-positive breast cancer patients were collected, which included age, body mass index (BMI), smoke, complications, ECOG PS score, LVEF, cardiac troponin I (cTnI), N-terminal (NT)-pro brain natriuretic peptide (BNP).

### Treatment

According to the National Comprehensive Cancer Network (NCCN) Clinical Practice Guidelines in Oncology for breast cancer (Version 4. 2017), at the preoperative period, patients received a trastuzumab-contained regimen (including AC → T (adriamycin plus cyclophosphamide followed by paclitaxel) + Trastuzumab, AC → D (adriamycin plus cyclophosphamide followed by docetaxel) + Trastuzumab, EC → T (epirubicin plus cyclophosphamide followed by paclitaxel) + Trastuzumab, and EC → D (epirubicin plus cyclophosphamide followed by docetaxel) + Trastuzumab and TC (docetaxel plus carboplatin) + Trastuzumab) as neoadjuvant treatment for 4–6 cycles, while in the postoperative period, patients continuously received trastuzumab therapy until the usage of trastuzumab up to 1 year as adjuvant treatment. Among these, 8 patients received AC → T + Trastuzumab, 10 patients received AC → D + Trastuzumab, 27 patients received EC → T + Trastuzumab, 37 patients received EC → D + Trastuzumab, and 15 patients received TC + Trastuzumab. Besides, 89 (91.8%) patients completed 1-year of adjuvant therapy.

### Samples Collection

Peripheral blood was extracted from breast cancer patients at baseline, after neoadjuvant treatment, at 3 months (M3), 6 months (M6), 9 months (M9), and 12 months (M12) after surgery. Immediately after each extraction, peripheral blood mononuclear cells (PBMC) and serum were isolated from the peripheral blood with a centrifuge by gradient centrifugation. Then, the PBMC was used for the detection of the expression of miR-497, and the serum was used for the detection of the level of FGF-23.

### miR-497 Detection

The relative expression of miR-497 was determined by reverse transcription-quantitative polymerase chain reaction (RT-qPCR). Total RNA was extracted by the RNeasy Protect Mini Kit (Qiagen, Duesseldorf, Germany), then 1 μg of total RNA was reverse-transcribed to cDNA using the PrimeScript RT reagent Kit (Perfect Real Time) (Takara, Dalian, China), and qPCR was carried out using SYBR Premix DimerEraser (Takara, Dalian, China). The design of primers for miR-497 referred to a previous report (18) as follows: miR-497, forward (5′->3′): ACACTCCAGCTGGGCAGCAGCACACTGTGG, reverse (5′->3′): TGTCGTGGAGTCGGCAATTC; U6 forward (5′->3′): CTCGCTTCGGCAGCACATATACTA, reverse (5′->3′): ACGAATTTGCGTGTCATCCTTGC. U6 was used as an internal reference. Relative quantification of gene expression was performed by the 2^−ΔΔCt^ method.

### FGF-23 Detection and miR-497/FGF-23 Axis Calculation

The level of FGF-23 in the serum was detected by enzyme-linked immunosorbent assay (ELISA) using the Human FGF23 ELISA Kit (Abcam, Shanghai, China). The procedure was in strict accordance with the instructions of the kit. After detection of the level of FGF-23, the miR-497/FGF-23 axis was calculated as the value of miR-497 expression divided by the value of the FGF-23 level according to a previous study (18).

### Cardiotoxicity Monitoring

For monitoring cardiotoxicity of the treatment, LVEF was measured using echocardiography at baseline, after neoadjuvant treatment, and at M3, M6, M9, and M12 after surgery. Meanwhile, the incidences of heart failure, acute coronary syndrome, and life-threatening arrhythmias were also recorded. The cardiotoxicity was defined as the occurrence of one of the following circumstances: (a) a change in the value of LVEF (ΔLVEF) from baseline ≥10% with the value of LVEF <53% simultaneously; (b) heart failure; (c) acute coronary syndrome; and (d) life-threatening arrhythmias.

### Statistical Analysis

SPSS 24.0 (IBM, Chicago, Illinois, USA) was used for statistical analysis. GraphPad Prism 8.01 (GraphPad Software Inc., San Diego, California, USA) was applied for graph plotting. Continuous variables were described as the mean ± standard deviation (SD) or median with interquartile range (IQR). Categorical variables were shown as counts with frequency. Comparations of repeated measures among different time points were determined by analysis of variance (ANOVA) or the Friedman test. Comparison of continuous variables between two groups was determined by the Wilcoxon sum rank test. Correlation analysis was determined by Spearman’s rank correlation test. A *p* value < 0.05 was considered statistically significant.

## Results

### Study Flow

Ninety-seven eligible patients received neoadjuvant trastuzumab plus chemotherapy, with blood samples being required before (baseline) and after neoadjuvant treatment. Then, patients received surgical resection; after that, blood samples were obtained at M3, M6, M9, and M12 after surgery during trastuzumab-involved adjuvant therapy. The blood samples were separated to get PBMCs and serum samples for detecting the miR-497 expression and FGF23 level, respectively (**Figure 1**).

**Figure 1:** Study flow chart.

### HER2-Positive Breast Cancer Patients’ Characteristics

The mean age was 51.9 ± 8.4 years, and there were 16 (16.5%), 14 (14.4%), 7 (7.2%), 17 (17.5%), and 8 (8.2%) patients complicated with hypertension, hyperlipidemia, diabetes mellitus, hyperuricemia, and chronic kidney disease, respectively. Besides, 77 (79.4%) patients were at 0 ECOG PS score and 20 (20.6%) patients were at 1 ECOG PS score. The mean value of LVEF was 66.4 ± 4.5. Furthermore, the median values of cTnI and NT-proBNP were 31.0 (11.0–65.0) pg/mL and 78.0 (63.5–107.5) ng/mL, respectively (Table 1).

**Table 1:** Characteristics of HER2-positive breast cancer patients.

Items	HER2-positive breast cancer patients (*N* = 97)
Age (years), mean ± SD	51.9 ± 8.4
BMI (kg/m^2^), mean ± SD	22.3 ± 2.2
Smoke, No. (%)	15 (15.5)
Hypertension, No. (%)	16 (16.5)
Hyperlipidemia, No. (%)	14 (14.4)
Diabetes mellitus, No. (%)	7 (7.2)
Hyperuricemia, No. (%)	17 (17.5)
Chronic kidney disease, No. (%)	8 (8.2)
ECOG PS score, No. (%)	
0	77 (79.4)
1	20 (20.6)
LVEF (%), mean ± SD	66.4 ± 4.5
cTnI (pg/mL), median (IQR)	31.0 (11.0–65.0)
NT-proBNP (ng/mL), median (IQR)	78.0 (63.5–107.5)

*SD, standard deviation; BMI, body mass index; ECOG, Eastern Cooperative Oncology Group; PS; performance status; LVEF, left ventricular ejection fraction; cTnI, cardiac troponin I; IQR, interquartile range; NT, N-terminal; BNP, brain natriuretic peptide.*

### Cardiotoxicity

LVEF was decreased from baseline to after neoadjuvant treatment and then at M3, M6, M9, and M12 after surgery (*p *< 0.001) (**Figure 2A**). Besides, the accumulating cardiotoxicity cases occurring after neoadjuvant treatment, at M3, M6, M9, and M12 after surgery were 2 (2.1%), 8 (8.2%), 15 (15.5%), 20 (20.6%), and 24 (24.7%), respectively (**Figure 2B**). In addition, the percentage of patients with total cardiotoxicity was 24.7%, among which the rate of patients with LVEF (ΔLVEF) from baseline ≥10% and the value of LVEF < 53%, heart failure, acute coronary syndrome, and life-threatening arrhythmias was 24.7%, 1.0%, 4.1%, and 0.0%, respectively (**Figure 2C**). Furthermore, among 24 patients who had cardiotoxicity events, 3 had relapsed and 1 died until the last follow-up date.

**Figure 2:** Cardiotoxicity events and incidences. Comparison of LVEF (**A**) and accumulating cardiotoxicity cases (**B**) among baseline, after neoadjuvant treatment, and at M3, M6, M9, and M12 after surgery. Percentage of patients with LVEF (ΔLVEF) from baseline ≥10% and the value of LVEF < 53%, heart failure, acute coronary syndrome, life-threatening arrhythmias, and total cardiotoxicity (**C**). Comparison of repeated measures among different time points was determined by analysis of variance (ANOVA).

### Changes in miR-497, FGF-23, and the miR-497/FGF-23 Axis among Different Time Points

MiR-497 expression was gradually decreased from baseline to M12 after surgery (*p *< 0.001) (**Figure 3A**), while FGF-23 expression was increased from baseline to M12 after surgery (*p *< 0.001) (**Figure 3B**). As for the miR-497/FGF-23 axis, it was persistently reduced from baseline to M12 after surgery (*p *< 0.001) (**Figure 3C**).

**Figure 3:** miR-497, FGF-23, and the miR-497/FGF-23 axis at different time points. Changes in miR-497 (**A**), FGF-23 (**B**), abs the miR-497/FGF-23 axis (**C**) among baseline, after neoadjuvant treatment, and at M3, M6, M9, and M12 after surgery. Comparison of repeated measures among different time points was determined by analysis of variance (ANOVA).

### Association of miR-497 with FGF-23 at Different Time Points

There was no correlation between miR-497 and FGF-23 at baseline (*p *= 0.104) (**Figure 4A**). However, miR-497 expression was negatively correlated with FGF-23 expression after neoadjuvant treatment (*p *= 0.003) (**Figure 4B**), at M3 after surgery (*p *< 0.001) (**Figure 4C**), at M6 after surgery (*p *< 0.001) (**Figure 4D**), at M9 after surgery (*p *< 0.001) (**Figure 4E**), and at M12 after surgery (*p *< 0.001) (**Figure 4F**).

**Figure 4:** Correlation of miR-497 with FGF-23 at different time points. Association of miR-497 with FGF-23 at baseline (**A**), after neoadjuvant treatment (**B**), and at M3 (**C**), M6 (**D**), M9 (**E**), and M12 (**F**) after surgery. Correlation analysis was determined by Spearman’s rank correlation test.

### Associations of miR-497, FGF-23, and the miR-497/FGF-23 Axis with Cardiotoxicity

MiR-497 was decreased in cardiotoxicity patients compared to noncardiotoxicity patients at M3 after surgery (*p *= 0.046), at M6 after surgery (*p *= 0.012), at M9 after surgery (*p *= 0.013), and at M12 after surgery (*p *= 0.005) (**Figure 5A**). As to FGF-23, it was increased in cardiotoxicity patients compared to noncardiotoxicity patients after neoadjuvant therapy (*p *= 0.047), at M3 after surgery (*p *= 0.011), at M6 after surgery (*p *= 0.004), and at M12 after surgery (*p *= 0.034) (**Figure 5B**). As for the miR-497/FGF-23 axis, it was reduced in cardiotoxicity patients compared to noncardiotoxicity patients at baseline (*p *= 0.042), after neoadjuvant therapy (*p *= 0.023), at M3 after surgery (*p *= 0.006), at M6 after surgery (*p *= 0.004), at M9 after surgery (*p *= 0.005), and at M12 after surgery (*p *= 0.002) (**Figure 5C**).

**Figure 5:** Comparison of miR-497, FGF-23, and the miR-497/FGF-23 axis between cardiotoxicity patients and noncardiotoxicity patients at different time points. Comparison of miR-497 (**A**), FGF-23 (**B**), and the miR-497/FGF-23 axis (**C**) between cardiotoxicity patients and noncardiotoxicity patients at baseline, after neoadjuvant treatment, and at M3, M6, M9, and M12 after surgery. Comparison of continuous variables between two groups was determined by the Wilcoxon sum rank test.

### Associations of miR-497, FGF-23, and the miR-497/FGF-23 Axis with LVEF

Regarding miR-497, it was positively correlated with LVEF at baseline (*p *= 0.005), after neoadjuvant therapy (*p *= 0.019), at M3 after surgery (*p *= 0.006), at M6 after surgery (*p *= 0.003), at M9 after surgery (*p *= 0.001), and at M12 after surgery (*p *< 0.001). As to FGF-23, it was negatively correlated with LVEF after neoadjuvant therapy (*p *= 0.035), at M3 after surgery (*p *= 0.001), at M6 after surgery (*p *= 0.014), and at M12 after surgery (*p *= 0.002). As for the miR-497/FGF-23 axis, it was positively associated with LVEF at baseline (*p *= 0.007), after neoadjuvant therapy (*p *= 0.006), at M3 after surgery (*p *< 0.001), at M6 after surgery (*p *= 0.002), at M9 after surgery (*p *= 0.002), and at M12 after surgery (*p *< 0.001) (Table 2).

**Table 2:** Correlation of miR-497, FGF-23, and the miR-497/FGF-23 axis with LVEF.

Items	Parameter	miR-497		FGF-23		miR-497/FGF-23 axis	
		*r*	*p* value	*r*	*p* value	*r*	*p* value
Time							
Baseline	LVEF	0.281	0.005	−0.062	0.549	0.271	0.007
After neoadjuvant therapy		0.238	0.019	−0.214	0.035	0.278	0.006
At M3 after surgery		0.279	0.006	−0.345	0.001	0.351	<0.001
At M6 after surgery		0.301	0.003	−0.248	0.014	0.316	0.002
At M9 after surgery		0.332	0.001	−0.118	0.250	0.304	0.002
At M12 after surgery		0.345	<0.001	−0.306	0.002	0.414	<0.001

*FGF-23, fibroblast growth factor-23; LVEF, left ventricular ejection fraction. The correlation analysis was performed by Spearman’s rank correlation test.*

### Association of miR-497, FGF-23, and the miR-497/FGF-23 Axis with Difference Treatment Regimens

There was no difference in miR-497, FGF-23, and the miR-497/FGF-23 axis among different treatment regimens at baseline, after neoadjuvant therapy, at M3 after surgery, at M6 after surgery, at M9 after surgery, and at M12 after surgery (all *p*’s* *> 0.05) (Supplementary Table S1).

## Discussion

Trastuzumab is the first approved monoclonal drug targeting the HER-2 gene for solid tumors, which is able to block the HER-2-mediated signal transduction pathway and accelerate the degradation of its receptor protein, subsequently decreasing the concentration of the cell membrane HER-2 protein, inhibiting angiogenesis, and killing tumors cells (19). Currently, trastuzumab has been used in the treatment of breast cancer with positive HER-2, and it improves the efficacy of chemotherapy and prolongs the progression-free survival of these patients (20). However, trastuzumab appears to be related to cardiotoxic reactions in breast cancer patients, and the most common clinical presentation is dilatation-hypokinetic cardiomyopathy, ten resulting in heart failure (8, 21, 22). In this study, we discovered that with the prolongation of trastuzumab-based neoadjuvant and adjuvant therapy in breast cancer patients, the level of LVEF continues to decline and the accumulating cardiotoxicity increases.

Although the detailed mechanisms of the trastuzumab-induced cardiotoxicity still remained unclear, the possible explanation was that trastuzumab intercepted neoreguline-1 (NRG-1)-mediated HER2 activation to inhibit fundamental intracellular mechanisms of cardiomyocytes (including the ability to maintain the structure and function of sarcomeres), subsequently causing the increase of accumulating cardiotoxicity in HER2-positive breast cancer patients (8, 23, 24).

MiR-497 has been clarified as a potential tumor suppressor in breast cancer (10–12, 25). For instance, an interesting study displays that miR-497 represses cell proliferation, promotes the percentage of early apoptotic cells, and suppresses G0/G1 cell phase arrest via targeting Bcl-w in breast cancer (10). Besides, miR-497 has been reported to be downregulated in human breast cancer cell lines compared to normal controls, and it inhibits cell colony formation and invasion by targeting Raf-1 (11). Furthermore, miR-497 also targets SMAD7 to decrease cell proliferation and invasion in breast cancer (12). Clinically, miR-497 expression was downregulated in breast cancer specimens compared to normal breast tissues, which is negatively associated with pathological stage, lymphatic metastasis, larger tumor size, and positive HER-2; also, its upregulation is correlated with better prognosis in breast cancer patients (10). In addition, miR-497 is inversely correlated with the malignancy of breast cancer patients (11). Interestingly, FGF-23 also has been reported to be involved in the pathological processes of breast cancer (13, 14). More importantly, miR-497 and FGF-23 have been found in several human organs and tissues (including heart and brain) (15–17), and miR-497 is implied in various cardiac pathogeneses (including mediating CDC differentiation through targeting the transforming growth factor beta signaling pathway (15) and promoting cardiomyocyte proliferation as well as inhibiting apoptosis by decreasing mitofusin 2 (Mfn2) expression in a mouse model of I/R injury (16)). In clinical, miR-497 expression has been discovered to be negatively correlated with the FGF-23 level, and the high level of the miR-497/FGF-23 axis is an independent predictive factor for lower accumulating MACCE occurrence in ESRD patients who underwent CAPD (18). Taken together, known that miR-497 and FGF-23 play roles in the pathogenesis of breast cancer, and the miR-497/FGF-23 axis is a predictive factor for cardiovascular and cerebrovascular events. Thus, we speculated that miR-497 might be correlated with trastuzumab-induced cardiotoxicity via interacting with FGF-23 in HER2-positive breast cancer patients treated with neoadjuvant treatment. In the present study, we found that with the prolongation of trastuzumab-based neoadjuvant therapy and adjuvant therapy time, miR-497 was gradually decreased, FGF-23 was gradually increased, and the miR-497/FGF-23 axis was gradually reduced in HER2-positive breast cancer patients.

More importantly, our results showed that the miR-497/FGF-23 axis had a better influence on responding to the cardiotoxicity of trastuzumab, which was stronger than miR-497 and FGF-23 alone in HER2-positive breast cancer patients. The possible explanations were that miR-497 not only accelerated cardiomyocyte proliferation and repressed inflammatory responses via targeting multiple genes (including mitofusin 2 and sirtuin 4) but also decreased FGF-23 to inhibit the local renin–angiotensin–aldosterone system, thereby repressing the cardiac hypertrophy and fibrosis in HER2-positive breast cancer patients. Therefore, the miR-497/FGF-23 axis had a better influence on responding to the cardiotoxicity of trastuzumab, which was stronger than miR-497 and FGF-23 alone.

Despite interesting findings in this study, some limitations still remained. The small sample size was the main limitation, which might lead to poor statistical power. Further validation in larger sample size is needed. Besides, this study was a single-center study, which might lead to selected bias. A further multicenter study is necessary. The third limitation was that the detailed mechanism of the miR-497/FGF-23 axis underlying trastuzumab-induced cardiotoxicity in breast cancer was not investigated. Further *in vivo* and *in vitro* experiments are needed.

In summary, the miR-497/FGF-23 axis may serve as a potential indicator predicting trastuzumab-induced cardiotoxicity in HER2-positive breast cancer patients.

## Data Availability

The original contributions presented in the study are included in the article/Supplementary Material; further inquiries can be directed to the corresponding author/s.
